# Effect of Intraoperative Ventilation Strategies on Postoperative Pulmonary Complications: A Meta-Analysis

**DOI:** 10.3389/fsurg.2021.728056

**Published:** 2021-10-04

**Authors:** Min Lei, Qi Bao, Huanyu Luo, Pengfei Huang, Junran Xie

**Affiliations:** Department of Anesthesiology, Sir Run Run Shaw Hospital of School of Medicine, Zhejiang University, Zhejiang, China

**Keywords:** low tidal volume ventilation, conventional mechanical ventilation, postoperative pulmonary complications, length of hospital stay, atelectasis

## Abstract

**Introduction:** The role of intraoperative ventilation strategies in subjects undergoing surgery is still contested. This meta-analysis study was performed to assess the relationship between the low tidal volumes strategy and conventional mechanical ventilation in subjects undergoing surgery.

**Methods:** A systematic literature search up to December 2020 was performed in OVID, Embase, Cochrane Library, PubMed, and Google scholar, and 28 studies including 11,846 subjects undergoing surgery at baseline and reporting a total of 2,638 receiving the low tidal volumes strategy and 3,632 receiving conventional mechanical ventilation, were found recording relationships between low tidal volumes strategy and conventional mechanical ventilation in subjects undergoing surgery. Odds ratio (OR) or mean difference (MD) with 95% confidence intervals (CIs) were calculated between the low tidal volumes strategy vs. conventional mechanical ventilation using dichotomous and continuous methods with a random or fixed-effect model.

**Results:** The low tidal volumes strategy during surgery was significantly related to a lower rate of postoperative pulmonary complications (OR, 0.60; 95% CI, 0.44–0.83, *p* < 0.001), aspiration pneumonitis (OR, 0.63; 95% CI, 0.46–0.86, *p* < 0.001), and pleural effusion (OR, 0.72; 95% CI, 0.56–0.92, *p* < 0.001) compared to conventional mechanical ventilation. However, the low tidal volumes strategy during surgery was not significantly correlated with length of hospital stay (MD, −0.48; 95% CI, −0.99–0.02, *p* = 0.06), short-term mortality (OR, 0.88; 95% CI, 0.70–1.10, *p* = 0.25), atelectasis (OR, 0.76; 95% CI, 0.57–1.01, *p* = 0.06), acute respiratory distress (OR, 1.06; 95% CI, 0.67–1.66, *p* = 0.81), pneumothorax (OR, 1.37; 95% CI, 0.88–2.15, *p* = 0.17), pulmonary edema (OR, 0.70; 95% CI, 0.38–1.26, *p* = 0.23), and pulmonary embolism (OR, 0.65; 95% CI, 0.26–1.60, *p* = 0.35) compared to conventional mechanical ventilation.

**Conclusions:** The low tidal volumes strategy during surgery may have an independent relationship with lower postoperative pulmonary complications, aspiration pneumonitis, and pleural effusion compared to conventional mechanical ventilation. This relationship encouraged us to recommend the low tidal volumes strategy during surgery to avoid any possible complications.

## What is Already Known About This Topic?

The role of intraoperative ventilation strategies in subjects undergoing surgery is still contested. This meta-analysis study was performed to assess the relationship between the low tidal volumes strategy and conventional mechanical ventilation in subjects undergoing surgery.

## What Does This Article Add?

The low tidal volumes strategy during surgery may have an independent relationship with lower postoperative pulmonary complications, aspiration pneumonitis, and pleural effusion compared to conventional mechanical ventilation.

This relationship encouraged us to recommend the low tidal volumes strategy during surgery to avoid any possible complications.

## Introduction

The harmful influence of intraoperative mechanical ventilation on subjects undergoing surgery under general anesthesia mainly includes ventilation-induced lung injury and postoperative pulmonary complications. The prevalence of postoperative pulmonary complications, a complex result of minor and major pulmonary complications, can reach up to 33% between the subjects undergoing surgery (1). Postoperative pulmonary complications have been reported to harm postoperative recovery by increasing the length of hospital stay, morbidity, and early mortality (2). The use of protective ventilation with low tidal volumes (4–8 ml/kg), a moderate level of positive end-expiratory pressure, and recruitment maneuvers have been suggested in intensive care unit patients with acute respiratory distress syndrome (3). However, the best intraoperative ventilation approaches for subjects undergoing surgery without severe lung injury remain unknown. Low tidal volume ventilation was related to improved pulmonary function than high tidal volume ventilation (4). However, conventional mechanical ventilation with high tidal volumes (more than 8 ml/kg) and little or no positive end-expiratory pressure (less than or equal to 5 cmH_2_O) without recruitment maneuvers is still recommended through general anesthesia (5). The present meta-analysis study aimed to find any possible relationship between the low tidal volumes strategy and conventional mechanical ventilation as intraoperative ventilation approaches in subjects undergoing surgery.

## Methods

The study performed here followed the meta-analysis of studies in the epidemiology statement (6), which was conducted following an established protocol.

### Study Selection

Included studies were those that reported statistical measures of relationship (odds ratio [OR], incidence rate ratio or relative risk, with 95% confidence intervals [CIs]) between the low tidal volumes strategy and conventional mechanical ventilation in subjects undergoing surgery.

Only human studies in any language were considered. Inclusion was not restricted by study size or publication type. Excluded publications were studies that did not provide a measure of a relationship. Figure 1 shows the whole study procedure.

**Figure 1:** Schematic diagram of the study procedure.

The articles were integrated into the meta-analysis when the following inclusion criteria were met:

1. The study was a randomized control trial or a retrospective study.
2. The target population included subjects undergoing surgery.
3. The intervention program had different intraoperative ventilation approaches.
4. The study included comparisons between the low tidal volumes strategy and conventional mechanical ventilation.

The exclusion criteria for the intervention groups were:

1. Studies that did not determine the effectiveness of intraoperative ventilation approaches in subjects undergoing surgery.
2. Studies that included the low tidal volumes strategy and conventional mechanical ventilation as intraoperative ventilation approaches in subjects undergoing surgery.
3. Studies that did not focus on the effect on comparative results.

### Identification

A protocol of search strategies was prepared according to the PICOS principle (7), and we defined it as follows: P (population): subjects undergoing surgery; I (intervention/exposure): intraoperative ventilation approaches; C (comparison): low tidal volumes strategy and conventional mechanical ventilation; O (outcome): postoperative pulmonary complications, length of hospital stay, atelectasis, aspiration pneumonitis, acute respiratory distress, short-term mortality, pneumothorax, pleural effusion, pulmonary edema, and pulmonary embolism; and S (study design): no restriction (8). First, we conducted a systematic search of OVID, Embase, Cochrane Library, PubMed, and Google scholar up to December 2020, using a combination of keywords and similar words for low tidal volume ventilation, conventional mechanical ventilation, postoperative pulmonary complications, length of hospital stay, atelectasis, aspiration pneumonitis, acute respiratory distress, short-term mortality, pneumothorax, pleural effusion, pulmonary edema, and pulmonary embolism as shown in Table 1. All identified studies were combined in an EndNote 16 file, duplicates were discarded, and the title and abstracts were reviewed to exclude studies that did not report a relationship between the low tidal volumes strategy and conventional mechanical ventilation in subjects undergoing surgery, based on the previously mentioned inclusion and exclusion criteria. The remaining articles were examined for correlated information.

**Table 1:** Search strategy for each database.

**Database**	**Search strategy**
Pubmed	#1 “low tidal volume ventilation”[MeSH Terms] OR “conventional mechanical ventilation”[All Fields] OR “postoperative pulmonary complications”[All Fields] #2 “length of hospital stay”[MeSH Terms] OR “low tidal volume ventilation”[All Fields] OR “atelectasis”[All Fields] OR “aspiration pneumonitis”[All Fields] OR “acute respiratory distress”[All Fields] OR “short-term mortality”[All Fields] OR “pneumothorax”[All Fields] OR “pleural effusion”[All Fields] OR “pulmonary edema”[All Fields] OR “pulmonary embolism”[All Fields] #3 #1 AND #2
Embase	'low tidal volume ventilation'/exp OR 'conventional mechanical ventilation'/exp OR 'postoperative pulmonary complications'/exp #2 'length of hospital stay'/exp OR 'atelectasis'/exp OR 'aspiration pneumonitis'/exp OR 'acute respiratory distress'/exp OR 'short-term mortality'/exp OR 'pneumothorax'/exp OR 'pleural effusion'/exp OR 'pulmonary edema'/exp OR 'pulmonary embolism'/exp #3 #1 AND #2
Cochrane library	#1 (low tidal volume ventilation):ti,ab,kw OR (conventional mechanical ventilation):ti,ab,kw OR (postoperative pulmonary complications):ti,ab,kw (Word variations have been searched) #2 (length of hospital stay):ti,ab,kw OR (atelectasis):ti,ab,kw OR (aspiration pneumonitis):ti,ab,kw OR (acute respiratory distress):ti,ab,kw OR (short-term mortality):ti,ab,kw OR (pneumothorax):ti,ab,kw OR (pleural effusion):ti,ab,kw OR pulmonary edema):ti,ab,kw OR (pulmonary embolism):ti,ab,kw (Word variations have been searched) #3 #1 AND #2

### Screening

Data were abridged based on study-associated and subject-associated features onto a consistent form: the last name of the primary author, period of study, year of publication, country, region of the studies, and study design; population type, the total number and the number of subjects undergoing surgery, demographic data, and clinical and treatment characteristics; operation type and method of assessment; result assessment; and statistical analysis OR or relative risk, along with 95% CI, of the relationship and its result (9). If a study qualified for inclusion based upon the aforementioned principles, data were extracted independently by two authors. In case of disagreement, the corresponding author provided a final opinion. When the data from a particular study differed based on the assessment of the relationship described above, we extracted the data separately. Individual studies were evaluated using the quality in prognosis studies tool, which evaluates validity and bias in studies of prognostic factors across six domains: participation, attrition, prognostic factor measurement, confounding measurement and account, outcome measurement, and analysis and reporting (10). Any inconsistencies were addressed by a re-evaluation of the original article.

The primary result concentrated on the low tidal volumes strategy and conventional mechanical ventilation in subjects undergoing surgery. A comparison between the low tidal volumes strategy and conventional mechanical ventilation was extracted to form a summary.

### Sensitivity and Subgroup Analyses

Sensitivity analyses were limited only to studies reporting the relationship between the low tidal volumes strategy and conventional mechanical ventilation in subjects undergoing surgery. For subgroup and sensitivity analyses, we used comparisons between the low tidal volumes strategy and conventional mechanical ventilation, as reference.

Dichotomous and continuous methods with a random or fixed-effect model were used to calculate the odds ratio (OR) or mean difference (MD) and 95% CI. We calculated the I^2^ index; the I^2^ index is between 0 and 100%. Values of approximately 0, 25, 50, and 75% indicate no, low, moderate, and high heterogeneity, respectively (11). When I^2^ was higher than 50%, we chose the random-effect model; when it was lower than 50%, we used the fixed-effect model. A subgroup analysis was performed by stratifying the original evaluation per outcome categories as described before. In this analysis, a *p*-value for differences between subgroups of <0.05 was considered statistically significant. Publication bias was evaluated quantitatively using the Egger regression test (publication bias considered present if *p* ≥ 0.05), and qualitatively, by visual examination of funnel plots of the logarithm of ORs or MDs vs. their standard error (SE) (7). All *p*-values were two-tailed. All calculations and graphs were performed using reviewer manager version 5.3 (The Nordic Cochrane Center, The Cochrane Collaboration, Copenhagen, Denmark).

## Results

A total of 3,421 unique studies were identified, of which 28 studies, from 2006 until 2020 in humans, satisfied the inclusion criteria and were included in the study (4, 12–38).

The 28 studies included 11,846 subjects undergoing surgery at baseline and reported a total of 2,638 receiving the low tidal volumes strategy and 3,632 receiving conventional mechanical ventilation. Those studies were to evaluate the relationship between the low tidal volumes strategy and conventional mechanical ventilation in subjects undergoing surgery. Fifteen studies reported that data were stratified in the ventilation strategy by postoperative pulmonary complications. Twenty-one studies reported that data were stratified in the intraoperative ventilation strategy by length of hospital stay; eleven studies by short-term mortality; sixteen studies by atelectasis; fourteen studies by aspiration pneumonitis; seven studies by acute respiratory distress; eight studies by pneumothorax; eight studies by pleural effusion; six studies by pulmonary edema; and four studies by pulmonary embolism as shown in Table 2.

**Table 2:** Characteristics of the selected studies for the meta-analysis.

**Study**	**Country**	**Total**	**Low tidal volume ventilation**	**Conventional mechanical ventilation**
Whalen et al. (12)	USA	20	10	10
Michelet et al. (13)	France	52	26	26
Cai et al. (14)	China	16	8	8
Weingarten et al. (15)	USA	40	20	20
Yang et al. (16)	South Korea	122	61	61
Ahn et al. (17)	South Korea	87	31	31
Treschan et al. (18)	Germany, Canada, and USA	395	50	51
Maslow et al. (19)	USA	34	17	17
Futier et al. (20)	France	1,803	200	200
Severgnini, et al. (21)	Italy	527	28	27
PROVE Network Investigators et al. (22)	Europe and North and South America	900	453	447
Fernandez-Bustamante et al. (23)	USA	28	14	14
Pi et al. (24)	China	63	20	22
Bolzan et al. (25)	Brazil	93	30	31
Park et al. (26)	South Korea	62	31	31
Wei et al. (27)	China	36	12	12
Aretha et al. (28)	Greece	122	45	45
Choi et al. (29)	South Korea	60	30	30
Pereira et al. (30)	Italy	40	20	20
Marret et al. (31)	France	346	172	171
Zhang et al. (32)	China	180	45	45
Soh et al. (33)	South Korea	97	39	39
Bluth et al. (4)	Europe and North and South America	2,013	1,002	1,011
Kim et al. (34)	South Korea	65	20	20
Li et al. (35)	China	472	126	126
Karalapillai et al. (36)	Australia	1,236	614	592
Cheng et al. (37)	Taiwan	68	30	29
Algera et al. (38)	Europe and North and South America	2,869	484	496
**Total**		**1,1846**	**3,638**	**3,632**

The study size ranged from 16 to 2,869 subjects undergoing surgery at baseline with 8 to 1,002 subjects receiving the low tidal volumes strategy, and 8 to 1,011 subjects receiving conventional mechanical ventilation. The low tidal volumes strategy during surgery was significantly related to a lower rate of postoperative pulmonary complications (OR, 0.60; 95% CI, 0.44-0.83, *p* < 0.001) with high heterogeneity (I^2^ = 76%), aspiration pneumonitis (OR, 0.63; 95% CI, 0.46-0.86, *p* < 0.001) with no heterogeneity (I^2^ = 0%), and pleural effusion (OR, 0.72; 95% CI, 0.56-0.92, *p* < 0.001) with low heterogeneity (I^2^ = 26%) compared to conventional mechanical ventilation as shown in Figures 2–4.

**Figure 2:** Forest plot of the low tidal volumes strategy vs. conventional mechanical ventilation in subjects undergoing surgery on postoperative pulmonary complications.

**Figure 3:** Forest plot of the low tidal volumes strategy vs. conventional mechanical ventilation in subjects undergoing surgery on length of hospital stay.

**Figure 4:** Forest plot of the low tidal volumes strategy vs. conventional mechanical ventilation in subjects undergoing surgery on short-term mortality.

However, the low tidal volumes strategy during surgery was not significantly correlated with length of hospital stay (MD, −0.48; 95% CI, −0.99–0.02, *p* = 0.06) with high heterogeneity (I^2^ = 91%); short-term mortality (OR, 0.88; 95% CI, 0.70-1.10, *p* = 0.25) with no heterogeneity (I^2^ = 0%); atelectasis (OR, 0.76; 95% CI, 0.57–1.01, *p* = 0.06) with no heterogeneity (I^2^ = 0%); acute respiratory distress (OR, 1.06; 95% CI, 0.67–1.66, *p* = 0.81) with low heterogeneity (I^2^ = 44%); pneumothorax (OR, 1.37; 95% CI, 0.88–2.15, *p* = 0.17) with no heterogeneity (I^2^ = 0%); pulmonary edema (OR, 0.70; 95% CI, 0.38–1.26, *p* = 0.23) with no heterogeneity (I^2^ = 0%); and pulmonary embolism (OR, 0.65; 95% CI, 0.26–1.60, *p* = 0.35) with no heterogeneity (I^2^ = 0%) compared to conventional mechanical ventilation as shown in Figures 5–11.

**Figure 5:** Forest plot of the low tidal volumes strategy vs. conventional mechanical ventilation in subjects undergoing surgery on atelectasis.

**Figure 6:** Forest plot of the low tidal volumes strategy vs. conventional mechanical ventilation in subjects undergoing surgery on aspiration pneumonitis.

**Figure 7:** Forest plot of the low tidal volumes strategy vs. conventional mechanical ventilation in subjects undergoing surgery on acute respiratory distress.

**Figure 8:** Forest plot of the low tidal volumes strategy vs. conventional mechanical ventilation in subjects undergoing surgery on pneumothorax.

**Figure 9:** Forest plot of the low tidal volumes strategy vs. conventional mechanical ventilation in subjects undergoing surgery on pleural effusion.

**Figure 10:** Forest plot of the low tidal volumes strategy vs. conventional mechanical ventilation in subjects undergoing surgery on pulmonary edema.

**Figure 11:** Forest plot of the low tidal volumes strategy vs. conventional mechanical ventilation in subjects undergoing surgery on pulmonary embolism.

A stratified analysis of studies that did and did not adjust for operation type, subjects' age, and ethnicities were not performed because not enough studies reported or adjusted for these factors.

Based on the visual inspection of the funnel plot as well as on quantitative measurement using the Egger regression test, there was no evidence of publication bias (*p* = 0.87).

## Discussion

This meta-analysis study based on 28 studies included 11,846 subjects undergoing surgery at baseline and reported a total of 2,638 receiving the low tidal volumes strategy and 3,632 receiving conventional mechanical ventilation (4, 12–38).

The low tidal volumes strategy during surgery was significantly related to a lower rate of postoperative pulmonary complications, aspiration pneumonitis, and pleural effusion compared to conventional mechanical ventilation.

The low tidal volumes strategy during surgery was not significantly correlated with length of hospital stay, short-term mortality, atelectasis, acute respiratory distress, pneumothorax, pulmonary edema, and pulmonary embolism compared to conventional mechanical ventilation. However, the length of hospital stay and atelectasis relationships had very low *p*-values (*p* = 0.06) suggesting that any added study may affect this insignificant result.

As shown from our meta-analysis results, low tidal volume is a very important piece of lung-protective ventilation. Though, according to the international expert-panel-based consensus recommendations on lung-protective ventilation for subjects undergoing surgery, not all ventilation approaches based on low tidal volumes result in lung protection (39). This could be because these outcomes are due to less pulmonary atelectasis, and better pulmonary compliance and oxygenation induced by moderate-to-high positive end-expiratory pressure (40, 41). Also, pneumoperitoneum through surgery may result in increased intrathoracic pressure, and decreased lung compliance and functional residual capacity (42). Recruitment maneuvers followed by subsequent moderate-to-high positive end-expiratory pressure are much more effective than positive end-expiratory pressure alone in re-expanding atelectasis and preserving the open dependent lung units (43).

Our finding is similar to that of a previous meta-analysis that reported a relationship between high-driving pressure and a high number of pulmonary complications (44). Atelectasis decreases lung compliance, and increases pulmonary vascular resistance and intrapulmonary shunting, causing the progression of postoperative pulmonary complications. In this study, the combination of low tidal volumes, moderate-to-high positive end-expiratory pressure, and recruitment maneuvers were better than conventional mechanical ventilation in decreasing the risk of atelectasis (44). Moderate to high levels of positive end-expiratory pressure can preserve end-expiratory lung volume, increase compliance, and consequently prevent atelectasis. Also, this influence could be stimulated by recruitment maneuvers, which overcome the opening pressure of the alveoli. A large cohort study even showed that low tidal volumes with minimal positive end-expiratory pressure were related to an increased risk of 30-day mortality (45). The use of high tidal volumes results in volutrauma, which injuries the alveolar, the vascular endothelial, the epithelial cells, and the extracellular matrix (46). This could activate an inflammatory response. Numerous randomized controlled trials have recommended that lung-protective ventilation strategies can reduce the release of inflammatory mediators (13, 47, 48). Also, animal studies reported that low tidal volumes ventilation with moderate-to-high positive end-expiratory pressure reduced bacterial growth in an experimental piglet model of pneumonia (49–51).

Two previous meta-analysis studies found a significant difference between protective ventilation and conventional ventilation in acute respiratory distress syndrome (52, 53). However, similar to our results another meta-analysis study did not find any significance in acute respiratory distress syndrome (54). The difference may be because of different methodologies used in those studies.

A stratified analysis of studies that did and did not adjust for operation type, subjects' age, and ethnicities were not performed because not enough studies reported or adjusted for these factors. However, from the study results presented here, we can recommend a low tidal volumes strategy during surgery to avoid any possible complications.

## Limitations

Some of the included articles were small in sample size, which has a potential risk of biases. There may be selection bias in this study since so many of the studies found were excluded from the meta-analysis. However, the studies excluded did not satisfy the inclusion criteria of our meta-analysis. A stratified analysis of studies that did and did not adjust for operation type, subjects' age, and ethnicities were not performed because not enough studies reported or adjusted for these factors. Some of the selected studies were retrospective, which might decrease the strength of fundamental evidence. Also, postoperative pulmonary complications were defined with considerable variation in the selected studies. Efforts at decreasing postoperative pulmonary complications mostly include postoperative ventilation strategies. Though, only a small number of the selected studies reported the ventilation strategies after surgery and the data were inadequate to perform an appropriate meta-analysis. Also, the subjects' enrollment strategies were not the same in the selected studies regarding inspiratory pressure, duration, and frequency.

## Conclusions

Based on this meta-analysis, the low tidal volumes strategy during surgery may have an independent relationship with lower postoperative pulmonary complications, aspiration pneumonitis, and pleural effusion compared to conventional mechanical ventilation. However, the low tidal volumes strategy during surgery was not significantly correlated with length of hospital stay, short-term mortality, atelectasis, acute respiratory distress, pneumothorax, pulmonary edema, and pulmonary embolism compared to conventional mechanical ventilation. This relationship encouraged us to recommend the low tidal volumes strategy during surgery to avoid any possible complications. However, further studies are needed to consolidate the beneficial effects of the ventilation strategy and to simplify the best levels of positive end-expiratory pressure, the best recruitment maneuver strategies, and the influence of postoperative ventilation strategies on clinical results.

## Data Availability Statement

The original contributions presented in the study are included in the article/Supplementary Material, further inquiries can be directed to the corresponding author/s.

## Author Contributions

JX: conception and design. ML, QB, HL, and PH: collection and assembly of data. All authors administrative support, provision of study materials or subjects, data analysis, interpretation, articles writing, final approval of manuscript, read, and approved the manuscript.

## Conflict of Interest

The authors declare that the research was conducted in the absence of any commercial or financial relationships that could be construed as a potential conflict of interest.

## Publisher's Note

All claims expressed in this article are solely those of the authors and do not necessarily represent those of their affiliated organizations, or those of the publisher, the editors and the reviewers. Any product that may be evaluated in this article, or claim that may be made by its manufacturer, is not guaranteed or endorsed by the publisher.
